The article "Importance of Gedunin in Antagonizing Rheumatoid Arthritis via Activating the Nrf2/ARE Signaling" was retracted in 2024. Reasons: signs of a paper mill; suspected computer-generated content; unreliable results or conclusions; concerns about the data.

# Importance of Gedunin in Antagonizing Rheumatoid Arthritis via Activating the Nrf2/ARE Signaling

**DOI:** 10.1155/2022/6277760

**Published:** 2022-04-07

**Authors:** Jian-Yu Chen, Xiao-Yun Tian, Wen-Jing Liu, Bao-Kun Wu, Yue-Chan Wu, Ming-Xing Zhu, Jin-Liu, Xian Zhou, Yan-Fang Zheng, Xue-Qin Ma, Ming-Qing Huang

**Affiliations:** ^1^Fujian University of Traditional Chinese Medicine, School of Pharmacy, Fuzhou, Fujian 350122, China; ^2^LiuHe Township Health Center, No. 63, LiuHe Road, Qi Chun Liu He, Huang Gang 436328, China; ^3^Fujian University of Traditional Chinese Medicine, Institute of Traditional Chinese Medicine, Fuzhou, Fujian 350122, China; ^4^NICM Health Research Institute, Western Sydney University, Penrith, NSW, Australia; ^5^Department of Pharmaceutical Analysis, School of Pharmacy, Key Laboratory of Hui Ethnic Medicine Modernization, Ministry of Education, Ningxia Medical University, Yinchuan, Ningxia 750004, China

## Abstract

**Objective:**

This study assessed the anti-arthritic effect and protection of Gedunin (GDN) on joint tissues and revealed the possible mechanism in suppressing rheumatoid arthritis (RA).

**Methods:**

LPS-induced macrophages and TNF-*α*-stimulated synovial fibroblasts (MH7A) or IL-1*β*-stimulated primary rheumatoid arthritis synovial fibroblasts (RASFs) were used to evaluate the antiinflammatory effect of GDN. In addition, CIA-induced arthritis was employed here to evaluate the anti-arthritic effect. MTT and BRDU assays were utilized to evaluate the cell viability and proliferation, Q-PCR was conducted to detect the mRNA expression of cytokines, FACS was adopted to monitor ROS production, while western blotting (WB) and siRNA interference were applied in confirming the anti-arthritic effects of GDN *via* the Nrf2 signaling. *Results. In vitro*, cell viability was inhibited in macrophages and MH7A cells, but not in RASFs; but the proliferation of RASFs was significantly suppressed in time- and dose-dependent manners. GDN suppressed cytokine levels in LPS-stimulated macrophages and TNF-*α*-stimulated MH7A cells or RASFs. GDN suppressed ROS expression. Furthermore, GDN treatment notably dose-dependently decreased the mRNA and protein expression of iNOS in LPS-induced macrophages. sip62 interference results showed that GDN cause the less expression of HO-1 and Keap1 and also fail to inhibit cytokines after sip62 interference. *In vivo*, GDN effectively inhibited paw swelling, arthritis score, and arthritis incidence and cytokines.

**Conclusions:**

Our study suggested that GDN exhibited strong antagonistic effect on arthritis both *in vitro* and *in vivo via* activation of Nrf2 signaling. Our work will provide a promising therapeutic strategy for RA.

The article "Importance of Gedunin in Antagonizing Rheumatoid Arthritis via Activating the Nrf2/ARE Signaling" was retracted in 2024. Reasons: signs of a paper mill; suspected computer-generated content; unreliable results or conclusions; concerns about the data.

## 1. Introduction

Rheumatoid arthritis (RA) is characterized by its high incidence all over the world. Actually, RA that involves inflammation and immunity usually results in redness, swelling, heat, and pain or even severe discomfort, disability, and death to some extent. The current therapeutics of RA have been greatly developed over the last decades, which can be mainly classified as four types, including nonsteroidal antiinflammatory drugs (NSAIDs), disease-modifying antirheumatic drugs (DMARDs), glucocorticosteroids, and antibodies of proinflammatory cytokines. However, these therapeutics show more or less side effects. Therefore, the current therapies should be further improved for their side effects.

A variety of cell populations are involved in RA pathogenesis, including macrophages, rheumatoid arthritis synovial fibroblasts (RASFs), T cells, and neutrophils. Among them, RASFs represent one of the most dominant cells existing in the terminal border lining of hyperplastic synovium, and they are located at the sites of adjacent cartilage and bone [1] [2] [3]. In normal individuals, only 1-3 cell layers, including RASFs and macrophages, exist from synovial border to joint cavity. However, in RA individuals, the lining thickness usually increases rapidly, and up to 10-15 cell layers may exist [4] [5] [6]. Subsequently, the intensive thickness of synovial lining, frequent influx, increased proliferation, and survival of RASFs may cause fierce synovial hyperplasia, which in turn induces inflammation in cells [1]. The severe synovial hyperplasia also provides a support for these synovial cells to attach to adjacent cartilage and bone through changing the expression of adhesion molecules [4] [5] [6]. In addition, RASFs not only produce various inflammatory cytokines, chemokines, proangiogenic factors, and matrix-degrading enzymes, but also form the proinflammatory milieu in the joints of RA patients, which is further involved in promoting inflammatory response and contributes to matrix degradation along with angiogenesis. All these results suggest that RASFs play important roles in the degradation of cartilage and bone in RA. Macrophages are another kind of important cells in inflammation and RA. Generally, macrophages are sensitive to numerous inflammatory stimuli, which can activate and produce inflammatory factors, nitric oxide (NO) and tumor necrosis factors when they are stimulated [7, 8]. The overexpression of inducible NOS (iNOS) and cyclooxygenase-2 (COX-2) will cause the release of NO and phenyl glycidyl ether (PGE), which in turn induces inflammatory responses [9]. Therefore, the cross-interaction between macrophages and RASFs results in RA initiation and severity.

The article "Importance of Gedunin in Antagonizing Rheumatoid Arthritis via Activating the Nrf2/ARE Signaling" was retracted in 2024. Reasons: signs of a paper mill; suspected computer-generated content; unreliable results or conclusions; concerns about the data.

The nuclear factor erythroid 2-related factor 2 (Nrf2) gene functions as a central antioxidative signaling in inflammatory or high oxidative stress (OS) events, such as reactive oxygen species (ROS) production, inflammatory cytokines, matrix metalloproteinases (MMPs), and chemokines secretion [10]. Nrf2 is involved in regulating the transcription of multiple genes, which is also reported to be associated with RA by restricting cartilage destruction and promoting the antioxidative signaling that results in antiinflammation [11–14]. More cartilage damages are observed in the joints of Nrf2 knockout arthritic mice [11]. In addition, the ROS levels increase in RA events [15][16], which can be resisted by the antioxidative signals, like Nrf2, thus inhibiting arthritis [14]. Dimethyl fumarate (DMF), which targets the Nrf2 pathway, was approved by FDA for the clinical treatment of multiple sclerosis (MS), which is another autoimmune disease. The latest report shows that DMF ameliorates complete Freund's adjuvant-induced arthritis in rats through the activation of the Nrf2/HO-1 signaling pathway [17]. Hence, Nrf2 serves as an important target for inflammation interference and OS of macrophages and RASFs in RA; therefore, it can be adopted as an effective therapeutic approach in the future.

Gedunin (GDN), a kind of limonoid isolated from natural sources, including *Azadirachta indica* (Meliaceae), is found to possess diverse biological activities, such as antimicrobial, antiinflammatory, and cytotoxic effects [18, 19]. It has been reported that GDN exerts its anti-allergic effect by modulating T cell activation [18]. Another study also observes that GDN has potent antiinflammatory and antinociceptive effects on the zymosan-induced inflamed knee joints [19]. In 2011, GDN has been first identified as an excellent candidate for high throughput screening of Nrf2 activators in Neh2-luciferase reporter assay [20]. As mentioned above, the activation of the Nrf2 signaling is closely involved in alleviating RA; hence, GDN may be a novel candidate for the effective suppression of RA. However, the effects of GDN against arthritis and the underlying mechanisms have not been reported so far. Therefore, this study was performed aiming to examine the anti-arthritic activity of GDN both *in vitro* and *in vivo*, so as to provide a novel support for the anti-RA drug discovery in preclinical settings.

## 2. Materials and Methods

### 2.1. Reagents

Macrophages (RAW264.7 cells) and MH7A cells were purchased from the American Type Culture Collection (ATCC, Manassas, VA, USA). The HepG2-C8 cell line was kindly presented by Prof. Ah-Ng Tony Kong from Rutgers University. The culture of RAW264.7, HepG2-C8, and MH7A cells was conducted according to our previous works [21, 22]. The primary RASFs were isolated from joint synovial cavity of RA patients, as described in our previous work [22]. The positive control, isoliquiritigenin (ILG) (purity, >98%, as verified by HPLC), was purchased from Nanjing Ze Lang Medical Technology Co., Ltd (Nanjing, China). Moreover, primary antibodies, including Keap1, Nrf2, HO-1, P-p62 (s349), and P-p62 (t269/s272) were obtained from Cell Signaling Technology (Boston, USA), whereas p62 and NQO1 were provided by ABcom (Cambridge, UK). The lipofectamine LTX kit was purchased from Invitrogen (Carlsbad, CA), while sip62 RNA and siRNA negative control (siRNA-NC) were obtained from Cell signaling technology (Boston, USA). Dulbecco's Modified Eagle's Medium (DMEM), OPTI-Minimum Essential Medium (MEM), fetal bovine serum (FBS), 100× penicillin-streptomycin (P/S), and Trypsin-EDTA (0.05%) were purchased from Gibco (Paisley, UK). Phosphate buffered saline (PBS), all primers, and the ROS/superoxide detection kit (DCFH-DA) were obtained from Invitrogen (Carlsbad, CA). 3-(4,5-dimethylthiazol-2-yl)-2,5-diphenyltetrazolium bromide (MTT), dimethylsulfoxide (DMSO), and methotrexate (MTX) were acquired from Sigma Aldrich (St. Louis, MI, USA).

The article "Importance of Gedunin in Antagonizing Rheumatoid Arthritis via Activating the Nrf2/ARE Signaling" was retracted in 2024. Reasons: signs of a paper mill; suspected computer-generated content; unreliable results or conclusions; concerns about the data.

### 2.2. MTT Assay

In brief, RAW 264.7 cells (5 × 10^3^/well) were seeded into the 96-well plates for 24 h and then treated with GND at various concentrations (0, 1, 2.5, 5, 10, 25, 50, and 100 *μ*M) for 24 h. MH7A cells (5 × 10^3^/well) were inoculated into the 96-well plates for 24 h and later exposed to GND treatment at various concentrations (0, 1, 5, 10, 25, 50, and 100 *μ*M) for 24 h. RASFs (5 × 10^3^/well) were seeded into the 96-well plates for 24 h and then treated with GND at various concentrations (0, 1, 5, 10, 25, 50, 100, and 150 *μ*M) for 24, 48, and 72 h, respectively. After incubation with GDN for anticipated hours, the cells were reacted with 5 mg/mL MTT for 4 h, respectively. Subsequently, the supernatant was removed carefully, and DMSO was added into the mixed solution within the 96-well plates to dissolve the purple precipitate under shaking for 15 min. Cell viability was detected in each well at 490 nm by an OD plate reader and is calculated by the following formula: cell viability (%) = OA_treated_/OA_control_.

### 2.3. Cell Proliferation Assay (BrdU Assay)

RASFs (5 × 10^3^/well) were seeded into the 96-well plates for 24 h and later treated with GDN at various concentrations (0, 1, 5, 10, 25, 50, 75, 100, and 150 *μ*M in RASFs) for 24, 48, and 72 h, respectively, following the cell proliferation assay protocol. Briefly, RASFs were labeled with BRDU (1×) at 16 h before they were harvested. Then, the labeling medium was removed through gentle tapping; the labeled cells were dried and incubated with 200 *μ*l/well FixDenat for 30 min at 15 °C-25 °C. Afterwards, the FixDenat solution was removed, and 100 *μ*l/well anti-BrdU-POD working solution was added to incubate for approximately 90 min at 15 °C-25 °C. Later, the antibody conjugate was eliminated by flicking off, and the wells were washed thrice with the 300 *μ*l/well washing solution. Thereafter, the 100 *μ*l/well substrate solution was added to incubate for 5-30 min at 15°C-25°Cuntil the color development was sufficient for photometric detection. Subsequently, the 1 M H_2_SO_4_ (25 *μ*l/well) was added into each well, and the microplate was incubated for about 1 min on the shaker at 300 rpm. Finally, the OD value was measured at 450/690 nm.

The article "Importance of Gedunin in Antagonizing Rheumatoid Arthritis via Activating the Nrf2/ARE Signaling" was retracted in 2024. Reasons: signs of a paper mill; suspected computer-generated content; unreliable results or conclusions; concerns about the data.

### 2.4. ROS Evaluation

To determine the impact of GDN on ROS, RASFs (2.5 × 10^5^/well) were treated with GDN at diverse concentrations (1, 5, 10, 25, and 50 *μ*M) for 48 h. After being washed with PBS once, the cells were collected by trypsin, rinsed with PBS, and stained with PBS containing 5 *μ*M DCFH-DA for 30 min. Subsequently, the DCFH-DA stained cells were collected by centrifugation at 1500 rpm, and the total ROS contents were analyzed using a FACScan flow cytometer.

### 2.5. Antioxidative Reaction Elements (ARE) Luciferase Reporter Activity Assay

To examine the effect of GDN on ARE, the HepG2-C8 cells stably transfected with the ARE-luciferase vector were used to perform the ARE luciferase assay according to our previous study [21].

### 2.6. Quantitative Reverse Transcriptase Polymerase Chain Reaction (qRT-PCR)

To detect the mRNA expression levels of iNOS, COX-2, IL-1*β*, TNF-*α*, IL-6, IL-33, HO-1, and NQO1, RAW264.7 cells (1 × 10^6^/well) were plated into the 6-well plates and preincubated with GDN at the concentrations of 1, 5, 10, and 25 *μ*M for 1 h. Then, the cells were stimulated by LPS (100 ng/ml) for another 24 h. To identify the mRNA expression levels of HO-1, NQO1, Nrf2, and p62, RAW264.7 cells (1×10^6^/well) and MH7A cells were treated with GDN at different concentrations for different time. To measure the mRNA expression levels of IL-1*β*, IL-6, and IL-33, MH7A cells were pretreated with GDN at anticipated concentration for 1 h and then incubated with TNF-*α* for additional 36 h. Moreover, to determine the IL-1*β* mRNA expression level in RASFs, RASFs were incubated for 1 h and then with TNF-*α* for another 24 h. The total RNA was extracted, and mRNA was quantified by qRT-PCR according to previous description [21].

The article "Importance of Gedunin in Antagonizing Rheumatoid Arthritis via Activating the Nrf2/ARE Signaling" was retracted in 2024. Reasons: signs of a paper mill; suspected computer-generated content; unreliable results or conclusions; concerns about the data.

### 2.7. Immunocytochemistry

To verify whether GDN induced the nuclear translocation of Nrf2, immunocytochemistry was performed on RASFs and RAW264.7 cells incubated with GDN at different concentrations. To be specific, RASFs (1 × 10^5^/well) and RAW264.7 cells (1 × 10^5^/well) were seeded onto the coverslips in the 6-well plates and incubated overnight, respectively, followed by 24 h of GDN treatments at different concentrations. Besides, the immunofluorescence cell staining was carried out according to our previous report [21].

### 2.8. Protein Extraction and Western Blotting (WB)

To investigate whether the expression of HO-1, NQO1, Keap1, p62, and Nrf2 was regulated by GDN, the cells were plated into the 6-well plates and treated with GDN at different concentrations for anticipated time. Then, the total cellular protein was extracted according to our previous work [21], separated by gel electrophoresis, and transferred onto the nitrocellulose membranes. Thereafter, the membranes were blocked with 5% free fat milk in the Tris-buffered saline 0.1% Tween 20 buffer and probed with specific antibodies.

### 2.9. siRNA Transfection

To verify whether GDN regulated the downstream signaling, siRNA interference was adopted to silence p62. In brief, MH7A (2 × 10^5^/well) cells were seeded into the 6-well plates overnight. Then, si-NC, sip62 (200 nM) and lipo2000 (3 *μ*l) were added into Opti-MEM to interfere with MH7A cells for 6 h. Subsequently, the original Opti-MEM was replaced with the fresh DMEM containing 20% FBS, cultured for 18 h, and incubated with GDN (50 *μ*M) for another 24 h, or GDN (50 *μ*M) for another 1 h and coincubated with TNF-*α* for another 36 h to verify whether GDN exert its antiinflammation through p62 signaling. Finally, the cellular protein and total RNA were harvested to evaluate the protein and mRNA.

### 2.10. Collagen-Induced Arthritis (CIA) in DBA Mice

The 8-week-old male DBA mice weighing 20-22 g were provided by Guangdong Medical Laboratory Animal Center. Then, DBA mice were fed with a standard diet ad libitum. The housing conditions (20 ± 0.5°C, 12/12 h light/dark cycle) were strictly monitored throughout the whole experiment. All *in vivo* experiments were approved by the Laboratory Animal Research Committee under the regulation of related guidelines.

Equal volumes of complete Freund's adjuvant and bovine type II collagen were added into a mortar to grind at a constant rate until its color changed from gray to white (the grinding time was normally no less than 30 min). The collagen was maintained on ice throughout the emulsification process. For obtaining the ideal arthritic model, DBA mice were immunized twice in total. Briefly, the tail and back near the tail of every mouse were cleaned and sterilized with 75% ethanol; then, for the first immunization, mouse back near the tail was intradermally injected with bovine CII emulsified in 0.1 ml CFA by a glass syringe. At 21 days later, the second immunization was carried out to achieve more intensive inflammatory response, and mice were subsequently injected with CII emulsified in 0.1 ml CFA. In this study, GND was dissolved into the solution consisting of physiological saline, PEG400 and DMSO (v/v, 6 : 3 : 1) to prepare the drug injection.

The article "Importance of Gedunin in Antagonizing Rheumatoid Arthritis via Activating the Nrf2/ARE Signaling" was retracted in 2024. Reasons: signs of a paper mill; suspected computer-generated content; unreliable results or conclusions; concerns about the data.

Moreover, the mice were randomly divided into 5 groups as follows. (1) Mouse in the Ctrl (normal) group were fed with a standard diet routinely throughout the experiment. (2) Mice in the model group were intraperitoneally administrated with solution in preparation every day. (3) Mice in the MTX group were intragastrically administered with 10 mg/kg/day and 0.2 ml/body MTX every 3 days. (4) Mice in the GDN group were given uniform intraperitoneal injection with GDN at different concentrations (2.5 and 5 mg/kg/day), as well as 0.2 ml/body on the day of second immunization, and the injections were given for 20 consecutive days until the termination of the experiment. The severity of arthritis was recorded every 2 days according to the arthritis score; in the meantime, hind paw thickness, incidence, and body weight were also measured. The arthritis score, which was determined by the severity of arthritis, was graded from 0 to 4 depending on the degrees of edema and erythema in periarticular tissues of each affected hind paw, where 0 = uninflamed, 1 = slight, 2 = moderate, and 3 = severe, and 4 = disability. Scoring was conducted by 2 independent observers who were blind to the experimental groups. In addition, hind paw thickness was measured using a Vernier caliper and presented as the mean thickness of both hind paws. Typically, the hind paw thickness was measured on the day of the second immunization, and the changes in hind paw thickness were calculated by subtracting the hind paw thickness measured on the day of the second immunization, which corresponded to the changes in body weight. The measurement was continued for about 20 days after the second immunization until the termination of the experiment.

### 2.11. Statistical Analysis

Data were presented as means ± SEM. One-way ANOVA with the Tukey's post hoc test in GraphPad Prism was adopted to analyze the significance of differences. ∗*p* < 0.05, ∗∗*p* < 0.01, and ∗∗∗*p* < 0.001 indicated that the differences were statistically significant vs control group, whereas ^#^*p* < 0.05, ^##^*p* < 0.01, and ^###^*p* < 0.001 declared statistically significant differences vs IL-1*β*, LPS, TNF-*α*, or model group.

The article "Importance of Gedunin in Antagonizing Rheumatoid Arthritis via Activating the Nrf2/ARE Signaling" was retracted in 2024. Reasons: signs of a paper mill; suspected computer-generated content; unreliable results or conclusions; concerns about the data.

## 3. Results

### 3.1. GDN Inhibited the Cell Viability of Macrophages and MH7A Cells and Suppressed the Proliferation of RASFs

In this study, the cell viability and proliferation of macrophages, MH7A cell, and RASFs were first detected by MTT and BrdU assays. According to our results, treatment with GDN at 50-100 *μΜ* for 72 h significantly induced the death of MH7A cells, and the cell death rate reached 99% at a concentration of 100 *μΜ* (Figure 1(c)). Additionally, as shown in Figure 1(d), GDN significantly reduced the cell viability of macrophages; to be specific, 25 *μ*M GDN suppressed cell viability by 26% compared with the vehicle-treated cells, while 55% cell viability was inhibited after treatment with 50 *μ*M GDN. After treatment with GDN at 100 *μ*M, the viability of up to 71% cells was suppressed. However, no visible cell death was observed under microscope after GDN treatments at the concentrations of 1, 5, 10, and 25 *μ*M (results not shown). By contrast, the cell viability of RASFs was almost insensitive to GDN treatment, even at the dose of 100 *μ*M for 24 h (Figure 1(a)). Furthermore, the cell viability of RASFs remarkably decreased in the presence of GDN at 48 and 72 h, respectively. Interestingly, GDN effectively inhibited the proliferation of RASFs in time- and dose-dependent manners, as exhibited in Figure 1(b). All these results showed that GDN significantly inhibited the cell viability of macrophages and MH7A cells in a dose-dependent manner, which also suppressed the proliferation of RASFs without killing them.

### 3.2. GDN Antagonized the Inflammatory Factors in Macrophages, MH7A Cells and RASFs, and Abolished ROS Production in RASFs

It is illustrated from Figures 2(a) and 2(b) that GDN significantly inhibited the iNOS mRNA (left) and protein expression (right); compared with LPS treatment alone, GDN effectively abolished the LPS-induced iNOS expression by about 90% at 10 *μ*M, and GDN treatment at 25 *μ*M induced almost the same mRNA expression as that in normal cells, which was consistent with WB results. In addition, the LPS-stimulated RAW 264.7 cells showed a markedly decreased expression of IL-1*β*, IL-6, and TNF-*α* after GDN treatment (Figures 2(c)–2(e)). Besides, GDN inhibited the mRNA expression of IL-1*β*, IL-6, and IL-33 in MH7A cells stimulated by TNF-*α* in a dose-dependent manner, as exhibited in Figures 2(f)–2(h).

However, only the expression of IL-1*β* was significantly reduced by GDN in TNF-*α*-stimulated RASFs, and MMP-13 production was suppressed in IL-1*β*-stimulated RASFs (Figures 2(i) and 2(j)). OS, in particular reactive oxygen species (ROS) production, accounts for a critical characteristic of RA, which has been abundantly found in joint diseases, such as osteoarthritis (OA) and RA [23]. ROS, including NO, peroxynitrite, and superoxide anion radicals, are involved in the synthesis and degradation of matrix components, finally resulting in cartilage degradation and joint inflammation [24]. Rationally, ROS production was evaluated by the FACScan flow cytometer, and the results demonstrated that GDN remarkably antagonized ROS production (Figures 2(k)–2(l)).

The article "Importance of Gedunin in Antagonizing Rheumatoid Arthritis via Activating the Nrf2/ARE Signaling" was retracted in 2024. Reasons: signs of a paper mill; suspected computer-generated content; unreliable results or conclusions; concerns about the data.

### 3.3. GDN Activated the Nrf2/ARE Signaling

As observed from Figure 3, GDN notably upregulated the mRNA expression of NQO1 and HO-1 in normal or LPS-stimulated macrophages, as presented in Figures 3(a) and 3(b) and 3(d)–3(e). Additionally, GDN also inhibited the protein expression of Keap1 and upregulated that of Nrf2 and HO-1 (Figures 3(c) and 3(f)). In MH7A cells, the mRNA expression levels of HO-1 and p62 were measured after GDN treatments for 1, 2, 4, 8, 12, and 24 h, respectively. As a result, the effect of GDN on activating the Nrf2 signaling peaked at 24 h, and GDN sharply increased the mRNA expression of p62 and HO-1 while remarkably upregulating that of NQO1 in time- and dose-dependent manners (Figures 3(j)–3(k)). Further WB results on the effect of GDN on MH7A cells also illuminated that GDN downregulated the expression of Keap1, but induced the expression of Nrf2, HO-1, NQO1, and p62 and phosphorylation of p62 (Figures 3(j)–3(k)) in the GDN-treated RASFs (Figures 3(l)–3(m)).

### 3.4. GDN Significantly Facilitated the Nuclear Translocation of Nrf2 and Activated the ARE Luciferase

As shown in Figures 4(a) and 4(b), the immunocytochemistry results demonstrated that GDN sharply increased the nuclear localization of Nrf2 in GDN-treated macrophages and RASFs. Further, nuclear extraction also indicated that GDN slightly increased the nuclear localization of Nrf2 and ameliorated its cytoplasmic localization (Figure 4(c)). It is well known that Nrf2 dimerizes the small Maf proteins and binds to ARE to activate the transcription of these antioxidant enzymes when it translocates to the cell nucleus [25]. Additionally, the activation of Nrf2 will cause increase in ARE. Therefore, we subsequently determined whether GDN promoted the ARE luciferase activity in HepG2-C8 cells stably transfected with the ARE-luciferase reporter vector. As shown in Figure 4(d), the reference compound, isoliquiritigenin (ILG), significantly enhanced the ARE luciferase activity, which was consistent with previous study [26]. As expected, GDN upregulated the ARE luciferase activity (Figure 4(d)). Collectively, these findings suggested that GDN promoted the nuclear translocation of Nrf2 in macrophages and RASFs, which in turn upregulated the transcription of antioxidative genes to inhibit inflammation.

The article "Importance of Gedunin in Antagonizing Rheumatoid Arthritis via Activating the Nrf2/ARE Signaling" was retracted in 2024. Reasons: signs of a paper mill; suspected computer-generated content; unreliable results or conclusions; concerns about the data.

### 3.5. Roles of Nrf2 and p62 in the GDN-Mediated anti-RA Signaling by Promoting anti-Oxidation

To validate whether GDN activated the Nrf2 signaling through p62, we first observed the effect of GDN on p62 mRNA and protein expression. As shown in Figure 3(i), we discovered that GDN amazingly raised the p62 mRNA and protein levels. Subsequently, we performed siRNA measurement in MH7A cells, the different results from those of negative group (NC) and sip62 group were obtained, illustrating that p62 expression was successfully reduced, as exhibited in Figure 4(e). However, GDN treatment did not reverse the sharp decrease in p62 protein expression after sip62 interference. Instead, the signaling from the p62 downstream, like Keap1 and HO-1, was successfully reversed after GDN treatment alone. Meanwhile, the diminished effects of GDN on IL-1*β*, IL-6, and IL-33 stimulated by TNF-*α* after sip62 interference were observed in our results (Figures 4(h)–4(j)).

### 3.6. GDN Postponed the Collagen-Induced Arthritis in DBA/1 Mice

It was demonstrated by the antiinflammatory study *in vitro* that GDN might inhibit RASFs proliferation, cytokine secretion, and ROS production, suggesting that GDN might possess excellent anti-RA effect. Here, we used bovine type II collagen and incomplete Freund's adjuvant to establish the CIA-induced arthritis model in DBA mice, which mimicked the clinical arthritic patients. Swelling of hind paws was regarded as a sign of arthritis onset and carefully examined every 2 days after the second immunization. The scoring of arthritis severity and arthritis incidence were also deemed as the indices of arthritis severity. As a result, swelling of hind paws was the most severe in CIA model than in other groups, while MTX and GDN treatments alleviated the swelling of hind paws. As shown in Figure 5(a), arthritis incidence in model group reached up to 83%, whereas MTX and GDN treatments delayed the onset of arthritis and decreased the arthritis incidence. It was observed from Figure 5 that the initial sign of slight swelling in hind paws occurred on around day 4 and paw swelling in mice with redness peaked on days 10-12. The swelling continued until day 14 in most mice and was gradually mitigated later. By contrast, mice injected with GDN showed a slight redness and swelling around the footpad. The severity of the above events in all arthritis mice decreased on day 14, even though cartilage tissue destruction still occurred. In addition, paw swelling, which peaked on around days 10-14, was gradually alleviated. These results illuminated that GDN treatment was essential for arthritis protection in this arthritis animal model. The results were shown as follows: Arthritis incidence, arthritis score, and paw edema are observed from Figures 5(b)–5(e), whereas bone erosion and bone volume are illustrated in Figure 6(a)–6(c). To evaluate the toxicity and side effect of GDN on the treatment of arthritis, we measure the mouse body weight after they were sacrificed at the end of the experiment. It is illustrated from Figure 5(f) that GDN failed to produce significant toxicity. Additionally, GDN significantly suppressed the mRNA expression of IL-1*β*.

The article "Importance of Gedunin in Antagonizing Rheumatoid Arthritis via Activating the Nrf2/ARE Signaling" was retracted in 2024. Reasons: signs of a paper mill; suspected computer-generated content; unreliable results or conclusions; concerns about the data.

## 4. Discussion

Rheumatoid arthritis (RA) is characterized by its high incidence all over the world. The current therapeutics of RA have been greatly developed over the last decades; however, there are a lot of problems in clinical practice; even if methotrexate (MTX) is the first-line treatment for RA, most patients are ineffective or intolerant. Therefore, reunderstanding RA pathogenesis, determining new therapeutic targets, and discovery for new therapeutic drugs based on these new targets will remain the focus of clinical medicine, biomedical science, and pharmaceutical science research in the future. Nrf2 signaling pathway can effectively protect against arthritic inflammatory diseases through diverse stages, such as regulating redox balance, detoxification, metabolism, and inflammation. Currently, dimethyl fumarate (DMF) targets the Nrf2 pathway and was approved by the FDA in 2013 for the clinical treatment of multiple sclerosis (MS), which is another autoimmune disease. Recent studies have shown that DMF can activate Nrf2 signaling to alleviate complete Fischer-adjuvant induced arthritis in rats [17], which reveal that Nrf2 pathway targets have become an important target for pharmaceutical researchers to develop anti-RA drugs.

We initially found that GDN had an intensive upregulated effect on HO-1, the downstream gene of Nrf2, which suggested that GDN might had the potential of anti-RA. Macrophages and RASFs, existing in the joint of arthritis, play important roles in RA pathogenesis. These two kinds of cells can secrete a series of inflammatory factors that are involved in arthritis development and inflammation monitoring. Therefore, we used two cell models, macrophages and RASFs, to verify the antiinflammatory effect of GDN *in vitro*.

MH7A cells are a kind of synovial fibroblasts isolated from RA patients, which are transfected with SV40 antigen to be the immortalized cells; therefore, they are similar to RASFs. Our results showed that GDN notably inhibited cell viability of macrophages and MH7A, but did not significantly decrease that of RASFs at 24 h. Additionally, no visualized cell death occurred in macrophages, and MH7A were detected. Then, we considered whether there was a possibility that GDN only inhibited cell proliferation but not cell viability. As demonstrated by BrdU assay results, GDN assuredly inhibited the proliferation of RASFs, suggesting that GDN suppressed RASFs proliferation but not cell viability in a short time; however, GDN effectively restrained RASFs proliferation and viability after 48 h. We speculated that the torpor characteristic of RASFs might be responsible for such result. Apart from this, GDN still blocked RASFs proliferation quickly and inhibited their cell viability persistently. Our results also indicated that MH7A cells were isolated from RA patients, but there was a significant difference in the sensitivity to chemical compounds. Thus, MH7A cells were only used as a reference in drug screening. Numerous chemokines are predicted to contribute to arthritis development because of their high expression levels in the synovial fluid of RA patients or in the arthritic paw of animal models [27]. Hence, the LPS-induced macrophages, TNF-*α*-stimulated RASFs, and MH7A cells were used in this study to mimic the inflammation and arthritis models. As a result, LPS activated the activities of iNOS, COX-2, IL-1*β*, IL-6, and TNF-*α*, which exhibited high expression levels in inflammation and arthritis to some extent. Also, we found that GDN successfully antagonized the mRNA expression of iNOS, IL-1*β*, IL-6, and TNF-*α*, suggesting that GDN might possess antiinflammation and anti-RA activities. We further evaluated the IL-1*β* mRNA expression in TNF-*α*-stimulated RASFs and discovered that GDN significantly inhibited IL-1*β*, but failed to inhibit IL-6 expression (data not shown). GDN also antagonized the MMP-13 mRNA expression in IL-1*β*-stimulated RASFs. Notably, the inhibition of these cytokines and MMPs provides a support for the anti-RA action.

The article "Importance of Gedunin in Antagonizing Rheumatoid Arthritis via Activating the Nrf2/ARE Signaling" was retracted in 2024. Reasons: signs of a paper mill; suspected computer-generated content; unreliable results or conclusions; concerns about the data.

Recent reports have revealed that both oxygen metabolism and inflammation occur in arthritis. To some extent, ROS, which are produced in the process of cellular oxidative phosphorylation, can aggravate OS [28]. Besides, the overproduction of ROS will damage proteins, lipids, nucleic acids, and matrix components, implying that ROS amplify the inflammatory response by regulating intracellular signaling molecules. Interestingly, our results showed that ROS were significantly downregulated by GDN. In addition, the ROS signaling results in Nrf2 activation, and HO-1 protects against the ROS-activated inflammation induced by TNF-*α*[29]. Nrf2 signaling has been identified as the upstream regulator of cytokine production [30]. Currently, the use of Nrf2 knockout mice can assist in exploring the relation between Nrf2 and arthritis. As found by an *in vivo* study, the mice of Nrf2 knockout group exhibit more severe cartilage injuries and more oxidative damage; meanwhile, the expression levels of Nrf2 target genes are higher in Nrf2-wild-type group than in the knockout group during the AIA-induced arthritis. Moreover, the amount of spontaneously fractured bones is observed in Nrf2 knockout mice with AIA stimulation [11]. Here, we also suspected whether GDN exerted the antiinflammatory or anti-RA effects through the activation of Nrf2. Then, we detected the mRNA and protein levels of antioxidative enzymes. As expected, GDN upregulated the mRNA expression of NQO1 and HO-1. Interestingly, further WB results also suggested that GDN promoted HO-1 expression and Nrf2 mRNA expression in RASFs and induced Nrf2 accumulation in these two cell lines, indicating that GDN probably prevented Nrf2 ubiquitination and promoted its expression. In addition, the increased HO-1 expression was attributed to Nrf2 activation; however, after shNrf2 treatment, GDN still upregulated HO-1 expression (data were not shown), which demonstrated that GDN activate HO-1 partly through Nrf2. Therefore, sip62 interference was performed to verify whether GDN exert its antiinflammatory effect through p62; we found that GDN failed to inhibit IL-1*β*, IL-6, and IL-33 stimulated by TNF-*α* after sip62 interference and demonstrated that the antiinflammatory effect of GDN is associated with p62.

Overall, the following conclusions were made according to the present work. (1) In macrophages, GDN significantly inhibited the cell viability of macrophages and suppresses iNOS expression in LPS-stimulated macrophages, but it had no impact on decreasing COX-2 expression (data not shown). Besides, IL-1*β*, IL-6, and TNF-*α* stimulated by LPS were antagonized by GDN treatment. (2) In fibroblasts, GDN inhibited MH7A cell viability, RASFs proliferation, ROS production in RASFs, and inflammatory factors (including IL-1*β*, IL-6, and IL-33), suggesting the antiinflammation potential of GDN. Typically, the antiinflammation effect was attributed to the upregulated antioxidative enzymes, like NQO1 and HO-1, which were regulated by Nrf2 activation through inhibiting Keap1 by inducing p62 expression. (3) *In vivo*, GDN significantly alleviated the CIA-induced arthritis in DBA/1 mice. The antiinflammatory and anti-arthritic effects and the underlying mechanisms of GDN are shown in Figure 6.

Our results also illustrated that p62 was possibly at a relatively upstream position in the complicated cross-talk signaling regulated by GDN. Furthermore, we explained the contribution of p62 to the activation of Nrf2 target genes in response to GDN treatment, which was to create a positive feedback loop by inhibiting Keap1 expression. These results provide convincing evidence that GDN contributes to suppressing OS in RASFs, which is a major requirement for limiting cartilage destruction. Further knowledge about the involvement of GDN in Nrf2 signaling may facilitate to develop novel therapeutic strategies for RA.

The article "Importance of Gedunin in Antagonizing Rheumatoid Arthritis via Activating the Nrf2/ARE Signaling" was retracted in 2024. Reasons: signs of a paper mill; suspected computer-generated content; unreliable results or conclusions; concerns about the data.

## Figures and Tables

**Figure 1:** Effect of GDN on macrophages and synovial fibroblasts viability and proliferation. (a, c-d) MTT assay of RASFs, MH7A cells, and macrophages in the presence of GDN at different doses and different time. (b) RASFs proliferation caused by GDN at different time point and doses. The cells were seeded into 96 well plates, and treatment with GDN at anticipated time and doses, MTT assay and cells proliferation were detected according to methods as we mentioned before. Values of ∗*p* < 0.05, ∗∗*p* < 0.01, and ∗∗∗*p* < 0.001 were declared statistically significant *vs* ctrl group.

**Figure 2:** Effect of GDN on inflammatory factors, MMPs, and ROS production in macrophages and synovial fibroblasts. (a-b) mRNA and protein levels of iNOS regulated by GDN in LPS-induced macrophages. (c-e) Inhibition of IL-1*β*, IL-6, and TNF-*α* mRNA expression by GDN in LPS-induced macrophages. (f-g) Antagonism of IL-1*β*, IL-6, and IL-33 mRNA levels by GDN in TNF-*α*-stimulated MH7A cells. (i-j) Influence of GDN on IL-1*β* and MMPs production. (k-l) Resistance of GDN to ROS production in RASFs. Cells were plated into 6 well plates and treated with GDN for optimized time and doses; cells total RNA and protein were collected for Q-PCR and western blotting, respectively. Living RASFs were harvested and dyed with DCFH-DA; then ROS was quantified by FACScan flow cytometer. Values of ∗*p* < 0.05, ∗∗*p* < 0.01, and ∗∗∗*p* < 0.001 were declared statistically significant vs ctrl group; ^#^*p* < 0.05, ^##^*p* < 0.01, and ^###^*p* < 0.001 were declared statistically significant *vs* IL-1*β* group, LPS group, or TNF-*α* group.

**Figure 3:** Effect of GDN on p62/Nrf2/HO-1 signaling pathway. (a-c) Activation of Nrf2 signaling by GDN in LPS-stimulated macrophages. (d-f) Activation of Nrf2 signaling by GDN in normal macrophages. (g-k) GDN activates p62/Nrf2/HO-1 signaling in MH7A cells in a time-dependent manner. (l-m) GDN caused Nrf2 activation in RASFs. Cells were seeded into 6 well plates and then treated with GDN for different time and different concentration. mRNA and protein were detected by Q-PCR and western blotting, respectively. Values of ∗*p* < 0.05, ∗∗*p* < 0.01, and ∗∗∗*p* < 0.001 were declared statistically significant vs control group; ^#^*p* < 0.05, ^##^*p* < 0.01, and ^###^*p* < 0.001 were declared statistically significant *vs* LPS group.

The article "Importance of Gedunin in Antagonizing Rheumatoid Arthritis via Activating the Nrf2/ARE Signaling" was retracted in 2024. Reasons: signs of a paper mill; suspected computer-generated content; unreliable results or conclusions; concerns about the data.

**Figure 4:** Effect of GDN on translocation of Nrf2 in macrophages and RASFs. (a) Induction of Nrf2 translocation induced by GDN in macrophages. (b-c) GDN increased Nrf2 translocation in RASFs. (d) Effect of GDN on ARE luciferase expression. (e-g) Expression of p62, HO-1, and Keap1 regulated by GDN after si p62 interference. (h-j) Expression of IL-1*β*, IL-6, and IL-33 stimulated by TNF-*α* after GDN treatment and sip62 interference. The cells were seeded into plates and handled by our previous methods; western blotting and immunocytochemistry assay were monitored for Nrf2 distribution; MH7A cells were seeded into 6 well plates, and then sip62 was performed according to the protocol; after sip62 treatment 36 h, GDN were coincubated for another 24 h; p62, Keap1, and HO-1 were detected by western blotting. Values of ∗*p* < 0.05, ∗∗*p* < 0.01, and ∗∗∗*p* < 0.001 were declared statistically significant vs control group or negative group.

**Figure 5:** Effect of GDN on collagen-induced arthritis in DBA/1 mice. (a) Procedure of collagen-induced arthritis and time point of treatment with GDN in CIA mice. (b) Images of representative paws from different groups. (c-f) Incidence of arthritis, hind paw swelling, arthritis score, and body weight in every group. (g) Micro-CT images of representative paws from different groups. (h-i) Influence of GDN on bone erosion and bone volume. (j-m) Inflammatory cytokines mRNA levels in every group. Values of ∗*p* < 0.05, ∗∗*p* < 0.01, and ∗∗∗*p* < 0.001 were declared statistically significant vs ctrl group; ^#^*p* < 0.05, ^##^*p* < 0.01, and ^###^*p* < 0.001 were declared statistically significant *vs* model group. After the second immunization with collagen until the terminal of experiment, mice were administered intraperitoneally with GDN 2.5, 5 mg/kg every day and intragastrically 10 mg/kg MTX every three days. Incidence of arthritis, hind paw swelling, arthritis score, and body weight in every group were recorded every two days.

**Figure 6:** GDN activates Nrf2 signaling to exert its antiinflammation and arthritis.

## Data Availability

The original data is available by contacting to corresponding authors.

## Abbreviations

ARE: Antioxidative reaction elements
CIA: Collagen-induced arthritis
COX-2: Cyclooxygenase-2
DCFH-DA: ROS/superoxide detection kit
DMARDs: Disease-modifying antirheumatic drugs
DMEM: Dulbecco's modified eagle's medium
DMF: Dimethyl fumarate
DMSO: Dimethylsulfoxide
FBS: Fetal bovine serum
GDN: Gedunin
ILG: Isoliquiritigenin
iNOS: Inducible NOS
MEM: OPTI-minimum essential medium
MH7A: TNF-*α*-stimulated synovial fibroblasts
MMPs: Matrix metalloproteinases
MS: Multiple sclerosis
MTT: 3-(4,5-dimethylthiazol-2-yl)-2,5-diphenyltetrazolium bromide
MTX: Methotrexate
NC: Negative group
NO: Nitric oxide
Nrf2: Nuclear factor erythroid 2-related factor 2
NSAIDs: Nonsteroidal antiinflammatory drugs
OA: Osteoarthritis
OS: Oxidative stress
P/S: Penicillin-streptomycin
PBS: Phosphate buffered saline
PGE: Phenyl glycidyl ether
qRT-PCR: Quantitative reverse transcriptase polymerase chain reaction
RA: Rheumatoid arthritis
RASFs: Rheumatoid arthritis synovial fibroblasts
ROS: Reactive oxygen species
siRNA-NC: siRNA negative control
WB: Western blotting.
